# Analysis of the Influence of Nursing Safety Management on Nursing Quality in Hemodialysis Room

**DOI:** 10.1155/2022/6327425

**Published:** 2022-07-16

**Authors:** Ying Huang, Hong Chen

**Affiliations:** Wuhan Blood Center, Wuhan, Hubei 430000, China

## Abstract

The influence of the nursing safety management in nursing quality of hemodialysis room was deeply analyzed through the evaluation index study of nursing quality in hemodialysis room. Sixty-two patients were selected from hemodialysis rooms as study samples, and 31 patients who had not carried out nursing safety management from September 2018 to September 2019 were selected as control samples. Thirty-one patients who underwent nursing safety management from September 2019 to September 2020 were included in the observation group. By comparing the samples of the control group and the observation group, it was found that the comprehensive score of adverse reaction risk nursing quality and nursing satisfaction score between the groups were significantly improved; *P* < 0.05. Nursing safety management can effectively reduce the quality of nursing in hemodialysis room and greatly reduce the occurrence of adverse risks.

## 1. Introduction

The main purpose of the hemodialysis room is to treat chronic renal failure, acute renal failure, refractory heart failure, cirrhosis, nephrotic syndrome, uremia, and other diseases. An important way to treat nephrosis is to exchange the vascular pathways and water in the patient's body, and drain the excess water in the patient's body through the process of dialyzer dialysis, membrane dialysis machine equipment, and toxin exchange, so as to finally maintain the water electrolyte balance and pH balance in the patient's body [1]. In this process, the nursing safety management of patients is particularly important, the nursing work in hemodialysis room is more intense than that of ordinary wards, and the nursing is more difficult. Nursing staff are required to have high professional skills to provide professional and high-quality services for hemodialysis patients.  Figure 1 shows the classification of blood loss during dialysis [2]. Therefore, it is very necessary to implement nursing safety management in hemodialysis room. This study aims to explore and analyze the impact of nursing safety management on nursing quality in hemodialysis room [3].

## 2. Literature Review

The nursing quality evaluation refers to the evaluation of the nursing quality and an objective conclusion through an organized and planned investigation and analysis of nursing activities according to relevant nursing management rules and standards [4]. The nursing quality evaluation is a systematic project, which consists of nursing quality evaluation organization evaluation way evaluation method evaluation index and evaluation standard. The nursing quality evaluation is an important part of nursing quality management, and the evaluation of hospital nursing quality is not only conducive to safeguarding the rights and interests of patients, and to ensure that patients get higher quality and safety of nursing services, but also to the hospital medical nursing work value affirmation. The evaluation can provide the basis for improving the quality of hospital medical care, and can also distinguish the advantages and disadvantages, so that the high-quality nursing service can be implemented and affirmed, and the inferior service can be punished and improved [5, 6]. The nursing quality evaluation is of great significance to nursing quality management. It can not only provide strong objective evidence for judging the current nursing quality, but also be conducive to continuous progress and survival in the fierce competition. It can measure the progress of nursing work, clarify the current level of nursing, further find the cause of the gap, correct the deviation, achieve the purpose of sustainable improvement of nursing quality, and ultimately ensure that patients get high-quality nursing services. The results of the nursing quality evaluation are also the embodiment of nursing work value and can prove the achievements of nursing work, so as to improve patient satisfaction and identification of nursing work, so as to promote the development of the nursing profession itself [7]. Laparoscopic radical prostatectomy (LRP) is the standard treatment for early-stage localized prostate cancer, of which urinary incontinence is the most common postoperative complication. Pelvic floor muscle rehabilitation training is recognized as a first-line intervention, but the existing rehabilitation training programs are not clear in the formulation process, the content is not uniform, and the clinical operability is not strong. In order to better guide the clinical rehabilitation of pelvic floor muscles after LRP and prevent urinary incontinence, Zheng et al. constructed a pelvic floor muscle rehabilitation training program for patients with LRP [8].

At present, there is still a certain gap between China's nursing quality management and that of hospitals in advanced countries. The nursing quality management system is not perfect and not effective enough. The evaluation of clinical nursing service quality is in the state of technical service mainly based on a technical operation under the traditional mode of paying attention to unified form and standardization of operation, and the management system does not adapt to professional development. The education and training of nursing managers in management knowledge are inadequate; in the aspect of human resource management quality control, there is the problem of a backward management system, which makes it difficult to continue to deepen the overall nursing. However, nursing quality standards are not updated enough, and some indicators are unscientific and lack indicators to reflect the changes in patients' health status. Quality inspection is popular in the form of examination, more nursing operations, less evaluation of the whole case, less evaluation of nurses' ability training, and even less evaluation of specialized nursing quality. The result is to highlight the details and neglect the content. The final inspection was highlighted, but the quality control was ignored, highlighting the specific technical operation, and ignoring the patient's physical and mental care. Individual indicators are highlighted, and the overall health outcomes of patients are neglected [9].

The nursing quality evaluation is a complicated and meticulous work. With the development of nursing science, the extension of nursing connotation and the content of clinical nursing quality evaluation are changing correspondingly. Some scholars divided the nursing quality evaluation into two parts: work quality index and work efficiency index. In the nursing quality control evaluation, the workload was taken into account, and the quantitative index of data-based management with quality priority and efficiency as the basic principle was determined. We propose that nursing performance evaluation should include the results of patients' nursing work and the impact of nursing work on the hospital, patient satisfaction, clinical nursing effect, and health education effect, as well as the impact of nursing quality on hospital image and economic benefits. The development and change of modern hospital service thought and quality idea make the nursing quality evaluation's view broader and broader. From life service technology service to psychosocial service, from technical effect to social benefit, from medical service use value to exchange value, from quality input to quality output, all have entered the evaluation range. In the patient-centered nursing service model, patient satisfaction survey is an important method to evaluate nursing quality.

In the nursing quality evaluation system, organizational structure construction is the basis and condition of quality assurance [10]. Outside China, some hospitals have special quality evaluation organizations, such as the Nursing Quality Assurance Committee, which is composed of nursing administrative staff, full-time nursing supervisors, instructors, head nurses, nursing educators, general nursing staff representatives, etc., with offices and staff to regularly evaluate the service quality [11, 12]. By establishing the quality control network structure of the head nurse of the nursing department and the head nurse of the department quality control group, and giving full play to the overall function of the three-level quality control management, the second-level comprehensive hospital in China has formed a strict self-control network and achieved optimized control effect. Total quality management requirements set a full clear guiding ideology and the full process of all the work, and the organization of the structure of nursing quality comprehensive management measures is to establish a mass quality control team, the nurse, acting through the involvement in quality control, strengthening quality consciousness, and consciously involved in quality improvement, and to constantly improve the quality of nursing service [13].

## 3. Study on Evaluation Index of Nursing Quality in Hemodialysis Room

### 3.1. Research Contents and Methods

The daily work in the hemodialysis room was recorded by status survey and semistructured interview, the process was standardized and modular, and the core important nursing items were determined to facilitate nursing management and quality evaluation, which was also the premise of this study [14]. Through clinical practice site investigation, a complete hemodialysis nursing process is included as follows:

① Patient preparation for dialysis: preparation of dialyzer and vascular access;
② Dialysis establishment: selection of parameters for blood circulation establishment by vascular puncture and system monitoring and treatment of dialysis complications; and
③ End of dialysis: feedback on the evaluation of patient withdrawal from dialysis [15].

All the above links can affect the dialysis effect and patients' satisfaction with dialysis services. Through the control of the dialysis process, medical staff constantly improve the dialysis methods, improve the dialysis effect, reduce dialysis complications, and improve the safety comfort, quality of life, and long-term survival rate of dialysis patients, which is the embodiment of dialysis quality management, and is also the quality management of dialysis center to achieve the goal [16, 17].

Due to the different roles of each evaluation index in the comprehensive evaluation, it is necessary to determine the weight coefficient of each evaluation index after determining the indicators of nursing quality evaluation, so as to ensure that the objectivity and rationality of the evaluation index standard determination of the impact of evaluation results are crucial. If the standard is too high, beyond the normal range and not in line with reality, it cannot play the role of the standard. If the standard is too low and the index changes are not sensitive, the discriminative validity of the evaluation results will be reduced and the induction and incentive effect of evaluation will be lost [18]. In this study, the weight and detailed rules of each index are determined through the status survey, expert consultation, and questionnaire survey, which are mainly used for the establishment of the weight coefficient of the consistency test of experts' opinions and the statistical analysis of each questionnaire.

### 3.2. Research Process

The research group was composed of 5 members, including a professor and graduate tutor, 2 clinical experts, and 2 graduate students. The research group was responsible for consulting data, formulating research topics, selecting consulting experts, preparing expert consulting tables, and analyzing and sorting out the consulting results [19].

Questionnaires were distributed and recovered by e-mail and on-site distribution of researchers. In the first round, two rounds of correspondence were conducted: alternative indicator pools and relevant background information were provided to experts. Comprehensive analysis and expert team, summary analysis results in the first round, and the second round of consultation questionnaire send experts in the same way. The first round to determine index connotation, according to the expert advice and index hoof pick standard index, increases or decreases for the second round of the final accord with standard indicators, using the expert sorting method to calculate each index weight value and one expert harmony coefficient. The second round of questionnaires was collected, and the expert opinions were comprehensively analyzed. The expert opinions basically tended to be the same. The letter consultation ended [20, 21].

The descriptive analysis of the index was expressed by the coefficient of variation of frequency constituent ratio mean standard deviation. The expert positive coefficient was expressed by questionnaire recovery rate. The degree of expert authority is expressed by the expert authority coefficient. The degree of concentration of expert opinions was expressed by the full mark ratio and the mean value of importance assignment. The degree of expert opinion coordination was expressed by the coefficient of variation and coefficient of expert harmony [22].

Excel data double entry to ensure accurate data entry and SPSS17.0 software were used for statistical analysis of data. According to the research purpose of this study and the theoretical research of previous relevant literature, the research route of this study is proposed, as shown in Figure 2.

### 3.3. Analysis of Research Results

According to statistics, important nursing items before dialysis in a hemodialysis room are as follows: evaluation of patients' nutritional status, patient's past history of infection, psychological status, vascular conditions, living habits, coagulation status, diet, patient's preparation, mood, mentality, target weight [23], and monitoring of patients' vital signs, especially blood pressure and temperature. The operation of the machine, especially the dialysis catheter in the pipeline, was observed to observe whether the preflushing of the machine was normal. Whether the vascular access is smooth, whether the vascular puncture site is red, swollen, hot, painful, whether there is infection, and whether there is weight gain.

The important nursing items in the hemodialysis room are as follows: monitoring the patient's vital signs and closely observing the reaction when dialysis, whether there is nausea, vomiting, sweating, muscle spasm, headache, dizziness, and other conditions; checking the machine operation, especially whether the parameter setting is accurate; and adjusting the parameters according to the doctor's advice. If the pipeline connection is tight, we patrol the patient and observe whether the puncture site is bleeding to observe whether the pipeline is unobstructed and whether the puncture site is bleeding to observe the nursing observation of the internal fistula catheter [24, 25].

The important nursing programs in the hemodialysis room are as follows: the nursing of fistula and catheter after dialysis, such as the compression and hemostasis of internal fistula, need to be guaranteed to be in good condition; if there is bleeding in arteriovenous fistula, the blockage needs to be removed after pressing; in addition, it also includes postoperative nursing and health education of internal fistula, such as using hot compress and massage, touching internal fistula everyday and every hour or so, and going to hospital for treatment in case of blockage.

For dietary care, it is necessary to control the intake of water and salt; evaluate whether the dialysis adequacy reaches the dry weight, accurately record the dry weight after dialysis, and prepare for the next dialysis; patients need to avoid drastic changes in vital signs, especially blood pressure. The positive coefficient of experts in this study was expressed as the ratio of experts participating in the evaluation to all experts by the questionnaire recovery rate, i.e.,

(1) $$\begin{array}{c} C_{j}=\frac{M_{j}}{M}. \end{array}$$

In the above formula, *C*_*j*_ represents the enthusiasm coefficient of experts; *M*_*j*_ represents the number of experts participating in the evaluation; and *M* represents total number of experts. The distribution and effective recovery of two rounds of questionnaires for all experts are shown in Table 1.

The expert consultation in this study invited nursing management and clinical experts from Grade-III, Grade-A hospitals, with a total of 30 people, the oldest of whom was 56 years old, and the youngest 32 years old, with an average of 42.53 and 5.022 years old, and other general information is shown in Table 2.

Table 2 shows that 70% of the experts have more than 10 years of nursing management experience, 60% of the experts have more than 5 years of dialysis experience, and all the experts have a bachelor's degree or above. About 60% of the experts have a title of head nurse or above, and 70% of the experts have a title of deputy director or above.

The authority of an expert (Cr) is generally determined by the basis on which the expert makes a judgment on the consultation content (Ca) and the expert's familiarity with the consultation content (Cs). The authority coefficient is equal to the arithmetic mean of the judgment coefficient and the familiarity coefficient. In general, prediction accuracy increases with the increase in expert authority.

The computational formula is as follows:

(2) $$\begin{array}{c} \text{Cr}=\frac{\left(\text{Ca}+\text{Cs}\right)}{2}. \end{array}$$

The expert judgment basis is divided into four categories: theoretical analysis, practical experience, reference to domestic and foreign materials, intuitive feeling, and the degree of influence that is divided into large, medium, and small, with corresponding assignment quantification, as shown in Table 3. Experts are divided into five levels of familiarity, such as very familiar, more familiar, generally less familiar, and less familiar, and the corresponding assigned value quantification, as shown in Table 4.

Judgment basis (Ca) is a comprehensive measure of the main factors upon which the expert makes a judgment on the question under investigation. The assignment of the degree of influence of expert judgment basis on expert judgment is shown in Table 4. This study provides the following questions in the judgment basis. We ask the experts to evaluate themselves. The self-assessment results are shown in Table 5.

It can be obtained from Table 5 that

(3) $$\begin{array}{c} \text{Ca}=\sum {\text{Ca}}_{i}\frac{m_{i}}{m},\\ =\frac{\left(\begin{array}{c} 0.3\times 19+0.2\times 10+0.1\times 1+0.5\times 24+0.4\times 4+0.3\times 2+\\ 0.1\times 5+0.05\times 16+0.05\times 9+0.1\times 2+0.07\times 12+0.05\times 16 \end{array}\right)}{30},\\ =0.869. \end{array}$$

Familiarity (*Cs*) is a measure of experts' familiarity with the investigated issues. The self-evaluation results of expert familiarity are calculated according to the contents of expert correspondence. See Table 6 for details.

According to the above data, the familiarity can be calculated as follows:

(4) $$\begin{array}{c} Cs=\left(1\times 7+0.8\times 21+0.6\times 2\right)/30=0.8333. \end{array}$$

The degree of expert authority (Cr) is as follows:

(5) $$\begin{array}{c} \text{Cr}=\left(\text{Ca}+\text{Cs}\right)/2=\left(0.869+0.8333\right)/2=0.8512. \end{array}$$

Generally speaking,

(6) $$\begin{array}{c} \text{Cr}\geq 0.70. \end{array}$$

When formula (6) is satisfied, the new capital is acceptable, and the *Cr* result of this study is 0.8512, indicating that the expert authority of this study is high and the result is credible.

The degree of concentration of expert opinions is represented by arithmetic mean and full score ratio. The larger the mean is, the higher the full score ratio is, and the more important the corresponding index is.

The degree of coordination of expert opinions is represented by the coefficient of variation of each item, also known as the standard difference rate, which is a statistical quantity to measure the degree of variation of each observed value in the data.

(7) $$\begin{array}{c} \text{CV}=\sigma /\mu . \end{array}$$

CV stands for coefficient of variation, *σ* stands for standard deviation, *μ* stands for arithmetic mean, and the smaller the coefficient of variation of arithmetic mean, the higher the coordination degree of experts, as shown in Table 7. Index hoof was selected according to the criteria of the mean value of importance assignment >3.00, the full score ratio >0.20, and the coefficient of variation <0.25. At the same time, combined with expert opinions, the results of index screening were determined after collective evaluation of the research group.

The results of the first round of expert letter consultation showed that the experts had no objection to the first-level indicators, and the proposed addition items of the second-level indicators were not accepted. The questionnaire for the proposed addition items of the three indicators and the detailed rules for modification were modified according to the expert opinions to form the second round of expert letter consultation table.

In the second round of expert consultation, experts were invited to compare and rank indicators at all levels, and the average rank of indicators with the same importance was taken. According to the rank assigned by experts to each indicator, the weight value of each indicator, the expert harmony coefficient, and the weight calculation formula of the difference test index were as follows:

(8) $$\begin{array}{c} \text{aj}=\frac{2\left[m\left(n+1\right)-\text{Rj}\right]}{\text{mn}\left(n+1\right)}, \end{array}$$

whereaj represents the weight of the *j*th indicator, *n* is the number of indicators, *m* is the number of experts, Rj represents the rank sum of the first indicator, and *W* is Kendall's harmony coefficient.

#### 3.3.1. The Calculation Formula of W When the Same Evaluator Does Not Have the Same Rating

(9) $$\begin{array}{c} W=\frac{S}{1/12K^{2}\left(N^{2}-N\right)}. \end{array}$$

*N* is the number of evaluated objects, *K* is the number of raters or the number of criteria on which the scores are based, and *S* is the sum of the ratings of each evaluated object *R*_*i*_ and the average of all these sums ${\bar{R}}_{i}$.

#### 3.3.2. The Calculation Formula of W When the Same Evaluator Has the Same Rating

(10) $$\begin{array}{c} W=\frac{S}{1/12\left[K^{2}\left(N^{2}-N\right)-K\sum_{i=1}^{k}T_{i}\right]}. \end{array}$$

Among them,

(11) $$\begin{array}{c} T_{i}={\sum_{i=1}^{m}\left(n_{\text{ij}}^{3}-n_{\text{ij}}\right)}^{2}. \end{array}$$

The significance test of Kendall's harmony coefficient is carried out according to the chi-square test criterion, and the formula is as follows:

(12) $$\begin{array}{c} x^{2}=k\left(n-1\right)w \end{array}$$

The degree of freedom formula is as follows:

(13) $$\begin{array}{c} \text{d}f=n-1. \end{array}$$

According to formula (13) and significance level *α*, the value *x*^2^ can be obtained from the value table *x*^2^. If it is greater than the value *x*^2^, it can be considered that the coordination coefficient is significant after the test, indicating that the expert opinion has good coordination and the result is desirable. Conversely, the smaller the value, the greater the probability of nonaccidental coordination of expert group opinions. Since the first round of expert consultation was completely back-to-back consultation and opinions were not communicated with each other by experts, the experts were not inspired by mutual opinions and could not explain the distribution of opinions after experts communicated with each other. Therefore, only the harmony coefficient of expert opinions and its significance test were analyzed for the second round of expert consultation, as shown in Table 8.

After the second round of expert letter consultation, the harmony coefficient of experts' opinions on the evaluation index system of nursing quality of hemodialysis room was statistically significant (*P* < 0.01) by significance test, indicating that all experts' opinions on the index system were coordinated; the next round of questionnaire was not issued; and the survey was ended.

## 4. Study on the Effect of Nursing Safety Management on Nursing Quality in Hemodialysis Room

### 4.1. Materials and Methods

General information is as follows: from September 2018 to September 2019, 31 patients treated with hemodialysis were selected as the control group without nursing safety management; from October 2019 to September 2020, 31 patients treated with hemodialysis were selected as the observation group with nursing safety management. In the observation group, there were 16 men and 15 women, aged 44–72 years old, with an average of (47.95 ± 4.86) years. In the control group, there were 17 men and 14 women, aged 44–74 years old, with a mean of (48.02 ± 4.87) years. The study was approved by the ethics committee of our hospital to compare the data of 62 hemodialysis patients, *P* > 0.05.

The control group carried out routine intervention, explained hemodialysis knowledge, gave psychological intervention combined with the psychological situation of patients, and carried out a basic nursing observation group to carry out nursing safety management, and the plan is as follows:

1. We determine the risk factors during hemodialysis, train the nursing staff on relevant knowledge, improve the daily nursing process, summarize the possible risk factors, and formulate solutions. In addition, we assign responsible nurses to check the daily nursing work and records.
2. We formulate emergency measures, including water and power failure in hemodialysis room, fire or hemodiaphoresis-related complications, etc. After formulating emergency measures, we carry out simulation drills and require nursing staff to respond calmly and timely.
3. We manage the related instruments in the hemodialysis room. Nursing staff in the hemodialysis room should master the models and the usage of all medical instruments, regularly check and maintain them, and strictly disinfect the instruments after use. In addition, responsible nurses should be arranged to record the use of the instrument and regularly maintain it to ensure the normal operation of the hemodialysis instrument. Meanwhile, the water treatment system should be overseen once every June to deal with abnormalities in the water system according to indexes such as residual chlorine water hardness and chemical pollution.
4. We manage the environment of the hemodialysis room, control the number of visitors entering the hemodialysis room every day, and reduce the contact between external personnel and hemodialysis patients, and medical staff entering and leaving the hemodialysis room should change clothes, wear special hats and gloves, and pay attention to hand hygiene. In addition, the hemodialysis room should be cleaned and regularly disinfected to regulate indoor temperature and humidity and improve patient comfort. For elderly hemodialysis patients, guardrails should be set up to reduce the risk of falling into bed.
5. We manage the patient's own risk factors and guide the patient to carry out relevant examinations to determine whether the patient is accompanied by infectious diseases before hemodialysis. For patients with blood-borne diseases, special dialysis machines should be selected for treatment, and responsible nurses should be assigned to care for them to reduce the risk of cross infection. In addition, during hemodialysis, needles should be properly fixed to reduce the risk of needle displacement and shedding.

The calculation software for hemodialysis patients was SPSS 33.0, the data recording index was%, $\bar{x}\pm s$, the statistical count measurement data was calculated, and the difference test between groups was performed in the form of *χ*^2^, *t*, *P* < 0.05, indicating statistically significant difference.

## 5. Results

The comparison of adverse reactions before and after nursing safety management is as follows: there were 6 cases of adverse reactions in the control group with an incidence of 19.35% and 1 case of adverse reactions in the observation group with an incidence of 3.23%, and the difference was statistically significant (*P* < 0.05), as shown in Table 9.

The comparison table of nursing quality and nursing satisfaction score between groups is as follows: after carrying out nursing safety management, nursing quality score and nursing satisfaction score in hemodialysis room were significantly improved. When comparing the data before nursing safety management, *P* < 0.05, as shown in Table 10.

## 6. Discussion

Hemodialysis rooms mainly treat patients with end-stage renal disease, and nursing staff perform hemodialysis operation according to medical advice. However, due to the high requirement of professional skills of nursing staff for hemodialysis operation, and the influence of patients' own factors and environmental factors, safety risks during hemodialysis are increased to a certain extent. Therefore, carrying out nursing safety management in hemodialysis room is of great significance to improve nursing quality. In the nursing safety management mode, the safety of hemodialysis can be improved by comprehensively evaluating risk factors during hemodialysis, developing targeted prevention and control programs, and strengthening the training of nursing staff to improve their professional skills and sense of responsibility. Improving relevant rules and regulations and urging nursing staff to carry out nursing operations according to the process can ensure the smooth operation of hemodialysis. Management of the hemodialysis room environment and regular disinfection of indoor temperature and humidity can improve the comfort of patients. Management of hemodialysis room instrument safety, thorough disinfection of patients' used instruments, and maintenance of normal operation of hemodialysis instruments can improve treatment efficiency and patient satisfaction. The risk of cross infection can be reduced by managing patient safety, controlling the number of people entering and leaving hemodialysis rooms, and determining whether patients have blood-borne diseases. Combined with the analysis of this study, after carrying out nursing safety management, the risk of adverse reactions is reduced, and nursing quality and nursing satisfaction score are increased, suggesting that nursing safety management has promotion value. In conclusion, the nursing safety management mode used in the nursing of hemodialysis patients can improve the nursing quality, reduce adverse risk events, and contribute to the harmonious nurse-patient relationship.

## 7. Conclusions

The hemodialysis room is the main place to treat chronic renal failure, acute renal failure, refractory heart failure, cirrhosis, nephrotic syndrome, uremia, and other diseases. The blood of the patient is guided through the vascular pathway through the dialysis membrane of the dialyzer device for water toxin exchange, so as to discharge the excess water in the body, maintain the water electrolyte balance and pH balance in the patient, and prolong the life of the patient. The hemodialysis room is an important place to carry out renal replacement therapy because of its special characteristics, strong professionalism, high requirements on the technical level of medical staff, large workload, and many emergencies. During the period of nursing intervention in the hemodialysis room, there are many hidden safety hazards, and medical disputes are very easy to occur, thus affecting the effect of dialysis. In recent years, the nursing safety management model has been gradually improved, which can be used in hemodialysis rooms to improve relevant systems on the basis of identifying hidden safety risks. Through the instrument environment and patient management models, the quality of nursing can be improved and the risk of adverse reactions can be reduced. Through nursing safety management, the nursing ability of nursing staff can be further improved, the safety risk prevention ability of nursing staff can be improved, the nursing quality of hemodialysis room can be further improved, and the nursing satisfaction of patients can be improved. Some studies have pointed out that the application of the nursing safety management in hemodialysis room can reduce the occurrence of nursing risk events and improve nursing satisfaction score. This study agrees with the above views. It can be seen from this study that nursing safety management attaches importance to adverse events' assessment of nursing safety management system and the overall nursing ability of nursing staff. By forming a group of nursing staff to study nursing safety consciousness, an intuitive and clear understanding of the blood dialysis room nursing safety, we set up a safety hazard prevention consciousness, effectively improve the nursing ability of nursing staff, constantly eliminate in blood dialysis room nursing safety, improve the security of hemodialysis patients, and further reduce the occurrence of nursing adverse events. The results of this study showed that compared with the control group that implemented conventional nursing management, the incidence of adverse nursing accidents in the experimental group that implemented nursing safety management was lower and the nursing quality score and nursing satisfaction score were higher. Therefore, the application of nursing safety management in hemodialysis room had significant effects.

## Figures and Tables

**Figure 1:** Classification of blood loss in dialysis.

**Figure 2:** Research technical route.

**Table 1:** Two rounds of expert correspondence questionnaire recycling.

	Number of releases (n)	Number of recycling (n)	Recovery rate (%)
First round	30	39	100
Second round	30	28	93.33

**Table 2:** General information on the 30 experts.

	Project	Number (n)	Composition ratio (%)
Age	Under 40 years of age	6	20.0
	40–50 years old	22	73.3
	Over 50 years old	2	6.7

Years of nursing management	Under 10 years	9	30.0
	10–15 years	13	43.3
	16–20 years	6	20.0
	More than 20 years	2	6.7

Years of dialysis service	Under 5 years	12	40.0
	5–10 years	11	36.7
	11–15 years	6	20.0
	More than 15 years	1	3.3

Degree	Master	2	6.7
	Undergraduate	28	93.3
	College and below	0	0.00

Office	Director of nursing	5	16.7
	Deputy director of nursing	6	20.0
	Sergeant major	7	23.3
	Nurse	12	40.0

Job title	Chief nurse	2	6.7
	Deputy chief nurse	19	63.3
	Nurse in charge	9	30.0

**Table 3:** The degree of influence of thirty expert judgment basis on expert judgment.

Judgment based	Influence degree of expert judgment			Influence degree of expert judgment
	Big	Middle	Small	
Theoretical analysis	0.30	0.20	0.10	
Experience	0.50	0.40	0.30	
Refer to domestic and foreign materials	0.10	0.08	0.05	
Intuitive feeling	0.10	0.07	0.05	
Total	1.00	0.75	0.50	

**Table 4:** Self-rated frequency of 30 experts' familiarity.

Familiarity	Very familiar	More familiar	Generally	Not familiar with	Unfamiliar
Expert self-assessment	1.0	0.8	0.6	0.4	0.2

**Table 5:** Thirty experts made their judgments based on self-rating frequency.

Judgment based	Big	Middle	Small
Theoretical analysis	19	10	1
Experience	24	4	2
Refer to domestic and foreign materials	5	16	9
Intuitive feeling	2	12	16

**Table 6:** Self-rated frequency of 30 experts' familiarity.

Project	Very familiar	More familiar	Generally	Not familiar with	Unfamiliar
Expert self-assessment	7	21	2	0	0

**Table 7:** Results of the first round of index expert letter consultation.

Metric name	Minimum	Maximum	Mean	Standard deviation	Coefficient	Full score ratio
I-1 Feature quality	1.00	5.00	3.9667	0.9279	0.2339	0.30
I-2 Link quality	3.00	5.00	4.5667	0.6261	0.1371	0.63
I-3 Terminal quality	3.00	5.00	4.2000	0.8052	0.1917	0.43
II-1 Environment, objects, and instruments△	3.00	5.00	4.0333	0.5561	0.1379	0.17
II-2 Human resource allocation	3.00	5.00	4.6667	0.6609	0.1416	0.77
II-3 Regulations	2.00	5.00	3.7000	0.9154	0.24 4	0.27
II-4 Disinfection and isolation	3.00	5.00	42333	0.7739	0.1828	0.43
II-5 Dialysis session	4.00	5.00	4.6667	0.4795	0.1027	0.67
II-6 Nursing session	3.00	5.00	3.8667	0.8604	0.2225	0.30
II-7 Quality of work	4.00	5.00	4.8667	0.3458	0.0710	0.87
II-8 Satisfaction	4.00	5.00	4.3667	0.4901	0.1122	0.37
III-1 Partition pass rate△	2.00	5.00	3.9667	0.9994	0.2520	0.37
III-2 Ward pass rate△	2.00	5.00	3.6000	0.8137	0.2260	0.13
III-3 Item pass rate△	2.00	5.00	3.4000	1.0034	0.2951	0.13
III-4 Instrument completeness	2.00	5.00	4.4000	1.0372	0.2357	0.70
III-5 Personnel qualification pass rate	1.00	5.00	3.7667	1.4065	0.3734	0.37
III-6 Staffing pass rate	1.00	5.00	4.0333	1.2452	0.3087	0.50
III-7 Management system improvement rate	3.00	5.00	4.0667	0.9072	0.2231	0.43
III-8 Improvement rate of diagnosis and treatment process and operation system	3.00	5.00	4.0667	0.6397	0.1573	0.23
III-9 Emergency plan improvement rate	2.00	5.00	4.2000	0.9248	0.2202	0.50
III-10 Hand hygiene pass rate△	1.00	5.00	3.7667	1.1351	0.3014	0.23
III-11 Instrument disinfection pass rate	2.00	5.00	4,2667	0.8683	0.2035	0.50
III-12 Pass rate for screening for blood-borne diseases△	1.00	5.00	3.9667	1.0662	0.2688	0.43
III-13 Water treatment system disinfection pass rate△	2.00	5.00	3.4667	1.1366	0.3279	0.27
III-14 Air purification pass rate	1.00	5.00	2.1333	1.3322	0.6245	0.07

Δ indicates the indicator that meets the criteria for deletion and modification.

**Table 8:** Expert opinion harmony coefficient and its significance test (*K* = 28).

Metric name	Number of entries	Coordination coefficient (W)	X^2^ value	Degree of freedom	*P* value
First-level indicator	3	0.2346	13.1376	2	<0.01
Secondary indicators	8	0.3424	67.1104	7	<0.01
Three-level indicators	30	0.3273	265.7676	29	<0.01

**Table 9:** Analysis of adverse reactions in hemodialysis room (case(%)).

Constituencies	Number of examples	Needle removal	Bleeding during dialysis	Infection	Incidence
Observation groups	31	1 (3.23)	0 (0.00)	0 (0.00)	1 (3.23)
Control group	31	3 (9.68)	1 (3.23)	2 (6.45)	6 (75.86)
x^2^					4.0260
P					<0.05

**Table 10:** Nursing quality and nursing satisfaction score analysis table (mark, $\bar{x}\pm s$).

Constituencies	Number of examples	Quality of care score	Nursing satisfaction rating
Observation groups	31	94.2 ± 6.35	91.19 ± 5.69
Control group	31	81.37 + 5.41	83.24 ± 4.31
T		8.6165	6.2011
P		<0.05	<0.05

## Data Availability

The labeled datasets used to support the findings of this study are available from the corresponding author upon request.

## References

[1] Djemiran D. (2020). Analysis performance of nursing personnel in inpatient room “darmayu” hospital ponorogo and the factors that influence. *JOURNAL FOR QUALITY IN PUBLIC HEALTH*.

[2] Zhang Q. L., Wang S., Zhang Y., Meng F. (2021). The effect of refined nursing intervention on patients undergoing maintenance hemodialysis in the hemodialysis center during the covid-19 epidemic. *BMC Nursing*.

[3] Shi-Fan, Han J.-L., Cheng Ya-P., Wang (2020). A bibliometric analysis of core articles of international nursing research frontiers based on the web of science database. *Frontiers of Nursing*.

[4] Straka L., Kuchta P. (2021). Analysis of the influence of tool electrode wear on surface quality in die-sinking edm technology. *MM Science Journal*.

[5] Yuan L., Yuan H., Feng Q., Zhao J. (2021). Effect of continuous nursing on quality of life of hemodialysis patients. *Medicine*.

[6] Thomas-Hawkins C., Flynn L., Dillon J. (2020). Registered nurse staffing, workload, and nursing care left undone, and their relationships to patient safety in hemodialysis units. *Nephrology Nursing Journal: Journal of the American Nephrology Nurses’ Association*.

[7] McGrath J. K., Elertson K. M., Morin T. (2020). Increasing patient safety in hemodialysis units by improving handoff communication. *Nephrology Nursing Journal*.

[8] Zheng Z. M., Hong B. Z., Mei E. N. (2022). Construction of pelvic floor muscle rehabilitation training program for patients undergoing laparoscopic radical prostatectomy. *Western Journal of Nursing Research*.

[9] Fauzi A., Triaswati R. (2021). The effect of intradialytic stretching training on restless legs syndrome and sleep quality in hemodialysis patients. *Korean Journal of Adult Nursing*.

[10] Sousa C. N., Marujo P., Teles P., Lira M. N., Dias V., Novais M. (2020). Self-care behavior profiles with arteriovenous fistula in hemodialysis patients. *Clinical Nursing Research*.

[11] Chae Y. J., Ahn J. H., Kang K. P., Jo E. (2020). Mediating effects of self-care competence on the relationship between uncertainty and quality of life in hemodialysis patients. *Korean Journal of Adult Nursing*.

[12] Yangz E. T., Zer Z. (2020). Nursing approach based on watson’s theory of human caring in treatment adherence in hemodialysis patients. *Bezmialem Science*.

[13] Aguiar L. L., Eloia S., Melo G., Silva R. A., Caetano J. F. (2020). Clinical judgment in nursing diagnoses of chronic kidney patients on hemodialysis. *Enfermería Global*.

[14] Mendes S., Pessoa N., Santos G., Niellys de Fátima da Conceio Gonalves Costa, Ramos V. P. (2020). Strategies to promote patient safety in hemodialysis: an integrative review. *Nephrology Nursing Journal: Journal of the American Nephrology Nurses’ Association*.

[15] Yu H., Meng Y., Li J., Shao S., Luo X. (2020). Evaluating effect of cognitive behavioral nursing on quality of life in hemodialysis patients. *American Journal of Internal Medicine*.

[16] Liu H., Li F., Liu F., Chen Y. (2020). Application of nursing quality index management in reducing the infection of tunnel-cuffed hemodialysis catheter. *Open Journal of Urology*.

[17] Song Y. Y., Chen L., Wang W. X., Yang D. J., Jiang X. L. (2022). Social support, sense of coherence, and self-management among hemodialysis patients. *Western Journal of Nursing Research*.

[18] Tan W. L., Khuan L., Baharom A., Arshad M. M. (2021). Coping strategies of patients with end stage kidney disease on hemodialysis: a systematic review. *Nephrology Nursing Journal: Journal of the American Nephrology Nurses’ Association*.

[19] Liu C., Lin M., Rauf H., Shareef S. (2021). Parameter simulation of multidimensional urban landscape design based on nonlinear theory. *Nonlinear Engineering*.

[20] Odom B., Elliott S., Barrios C. G. (2021). Promoting patient and nurse safety in acute dialysis units through advocacy and collaboration. *Nephrology Nursing Journal*.

[21] Nazly E., Khatib H. A. (2021). The knowledge and educational needs of nurses regarding pain management of patients on maintenance hemodialysis: a qualitative study. *The Open Nursing Journal*.

[22] Dogra J., Jain S., Sharma A., Sood M. (2020). Brain tumor detection from MR images employing fuzzy graph cut technique. *Recent Advances in Computer Science and Communications*.

[23] Balakrishnan N., Rajendran A., Ajay P. (2021). Deep embedded median clustering for routing misbehaviour and attacks detection in ad-hoc networks. *Ad Hoc Networks*.

[24] Liu X., Liu J., Chen J., Zhong F. (2022). Degradation of benzene, toluene, and xylene with high gaseous hourly space velocity by double dielectric barrier discharge combined with Mn3O4/activated carbon fibers. *Journal of Physics D: Applied Physics*.

[25] Huang R., Yan P., Yang X. (2021). Knowledge map visualization of technology hotspots and development trends in China’s textile manufacturing industry. *IET Collaborative Intelligent Manufacturing*.

